# Correlation of Platelet Function with Postpartum Hemorrhage and Venous Thromboembolism in Patients with Gestational Hypertension Complicated with Diabetes

**DOI:** 10.1155/2022/2423333

**Published:** 2022-07-18

**Authors:** Nan Li, Yang Liu, Anqi Yun, Shurong Song

**Affiliations:** ^1^Department of Obstetrics, The Third Central Hospital of Tianjin, 83 Jintang Road, Hedong District, Tianjin 300170, China; ^2^Department of Obstetrics, Tianjin Key Laboratory of Extracorporeal Life Support for Critical Diseases, Tianjin 300170, China; ^3^Department of Obstetrics, Artificial Cell Engineering Technology Research Center, Tianjin 300170, China; ^4^Department of Obstetrics, Tianjin Institute of Hepatobiliary Disease, Tianjin 300170, China

## Abstract

**Objective:**

This study was aimed at investigating the correlation of platelet function with postpartum hemorrhage and venous thromboembolism (VTE) in gestational hypertension patients with diabetes mellitus.

**Methods:**

A total of 93 patients with gestational hypertension complicated with diabetes treated from March 2020 to June 2021 were selected as the research group, and 56 healthy pregnant women during the same period were selected as the control group. Platelet function-related indicators (platelet count (PLT), platelet volume distribution width (PDW), and mean platelet volume (MPV)) were compared between the two groups. The patients were divided into a severe group (*n* = 13), mild group (*n* = 28), and nonbleeding group (*n* = 52) according to the severity of postpartum hemorrhage, and the value of combined detection of platelet function-related indicators on the severity of postpartum hemorrhage was evaluated and analyzed. According to the occurrence of VTE, the patients were divided into a VTE group and non-VTE group to analyze the predictive value of combined detection of platelet function-related indicators for VTE occurrence in patients.

**Results:**

The PLT value of the study group was lower than that of the control group, while the PDW and MPV values were higher than those of the control group (all *P* < 0.05). The PLT value increased with the aggravation of postpartum hemorrhage, while the PDW and MPV values decreased with the aggravation of postpartum hemorrhage among the three groups with different severities of postpartum hemorrhage (all *P* < 0.05). The area under the curve (AUC) of PLT, PDW, and MPV combination to evaluate the severity of postpartum hemorrhage in patients with gestational hypertension combined with diabetes was greater than that of PLT alone and PDW alone (both *P* < 0.05). The PLT value was negatively correlated with the severity of postpartum hemorrhage, while PDW and MPV values were positively correlated with the severity of postpartum hemorrhage (both *P* < 0.05). According to the occurrence of VTE, patients were divided into the VTE group (*n* = 10) and non-VTE group (*n* = 83). The PLT value of the VTE group was higher than that of the non-VTE group, while the PDW and MPV values were lower than those of the non-VTE group (all *P* < 0.05). The AUC of PLT, PDW, and MPV combination to predict the occurrence of VTE in patients with gestational hypertension combined with diabetes was greater than that of each index alone (all *P* < 0.05).

**Conclusion:**

Patients with gestational hypertension complicated with diabetes had abnormal platelet function, and the platelet function was related to postpartum hemorrhage and VTE.

## 1. Introduction

During pregnancy, the body will undergo a series of adaptive physiological and biochemical changes, which are mainly manifested in the gradual tendency of blood to hypercoagulability in hematology [1]. Gestational hypertension, as a pregnancy-specific disease, is the main factor affecting maternal and infant health and the main cause of maternal and perinatal mortality and morbidity [2]. It has been reported that thrombocytopenia and abnormal coagulation function play an important role in the occurrence and development of gestational hypertension [3]. Other studies have pointed out that pregnant women with hypertension during pregnancy have evident blood hypercoagulability and significantly higher incidence of thrombosis than normal pregnancy. Postpartum hemorrhage is a serious complication of hypertension during pregnancy and an important factor leading to maternal death [4]. Gestational diabetes mellitus (GDM) is a common complication of pregnancy. It refers to the abnormality of glucose metabolism first discovered or occurring during pregnancy. Zhang et al. [5] reported that platelet activation and coagulation activity in patients with GDM significantly increased, and changes in platelet function indicators seriously affect pregnancy outcomes. Diabetes can damage the blood vessel endothelial nuclear anticoagulant system, promote the activation of platelets and blood coagulation system, and then cause the blood to present the prethrombotic state or even form thrombus in severe cases. Other studies have found that maternal blood will undergo a series of changes during pregnancy, with increased contents of thrombin, coagulation factors, and fibrinogen in blood, weakened anticoagulant and fibrinolytic functions, and blood presenting a state of hypercoagulation; thus, the probability of venous thromboembolism (VTE) will be greatly increased [6]. Postpartum hemorrhage is a serious obstetric complication and the leading cause of maternal death in China. As the blood of pregnant women is in a high coagulation state, postpartum hemorrhage is prone to cause diffuse intravascular coagulation, which ultimately leads to the occurrence of multiple organ dysfunction syndrome. Relevant reports indicate that pregnant women with risk factors such as pregnancy complications are more likely to suffer from postpartum hemorrhage [7]. However, no report has clearly indicated the relationship between platelet function and postpartum hemorrhage as well as VTE occurrence in patients with gestational hypertension complicated with diabetes. Therefore, correlation analysis was conducted in this study to provide reference for the evaluation and clinical prognosis prediction of the disease.

## 2. Data and Methods

### 2.1. Clinical Data

A total of 93 patients with gestational hypertension complicated with diabetes from March 2020 to June 2021 were selected as the research group, which met the diagnostic criteria of gestational hypertension and GDM in relevant guidelines [8, 9]. Gestational hypertension: hypertension first appeared after 20 weeks of pregnancy, systolic blood pressure was ≥140 mmHg and/or diastolic blood pressure was ≥90 mmHg but returned to normal within 12 weeks after delivery, and the urine protein test was negative. GDM: (1) oral glucose tolerance test (OGTT) was 75 g, and glucose value of fasting and 1 h and 2 h after taking glucose should not exceed 5.1 mmol/L, 10.0 mmol/L, and 8.5 mmol/L, respectively; GDM is diagnosed if there is one abnormality in 3 times. (2) Fasting blood glucose ≥ 5.1 mmol/L at 24-28 weeks was directly diagnosed as GDM. If fasting blood glucose ≥ 4.4 mmol/L and <5.1 mmol/L, OGTT shall be performed for definite diagnosis. Pregestational diabetes mellitus (PGDM) was diagnosed when fasting blood glucose in early pregnancy was ≥7.0 mmol/L, OGTT 2 h was ≥11.1 mmol/L, or random blood glucose was ≥11.1 mmol/L. A total of 56 healthy pregnant women were selected as the control group. There was no significant difference in general data between the two groups (*P* > 0.05, Table 1). We passed the ethics review in August 2021. Before enrollment, we informed patients of the purpose and process of the experiment and obtained informed consent from patients.

### 2.2. Inclusion Criteria

The inclusion criteria were as follows: (1) complete clinical data, (2) those who have not taken drugs affecting platelet and coagulation function in the last 3 weeks, and (3) single pregnancy.

### 2.3. Exclusion Criteria

Exclusion criteria were as follows: (1) patients with autoimmune diseases, (2) patients with blood system diseases, (3) patients with essential hypertension, (4) diabetes appearing before pregnancy, (5) patients with malignant tumor, (6) patients with severe liver and kidney dysfunction, (7) patients with infectious diseases, and (8) patients with serious cardiovascular and cerebrovascular diseases.

### 2.4. Methods

#### 2.4.1. Platelet Function Test

On the day of enrollment, 3 mL of fasting venous blood was collected from the subjects, and the platelet count (PLT), platelet distribution width (PDW), and mean platelet volume (MPV) of the patients were detected with a SYSMEX five-category hematology analyzer (XE-5000).

#### 2.4.2. Severity of Postpartum Hemorrhage

Severity of postpartum hemorrhage in the study group was evaluated by referring to *Guidelines for Prevention and Management of Postpartum Hemorrhage (2014)* [10]: postpartum hemorrhage: blood loss in vaginal delivery ≥ 500 mL or blood loss in cesarean delivery ≥ 1000 mL, and severe postpartum hemorrhage: blood loss ≥ 1000 mL within 24 h after delivery.

#### 2.4.3. VTE Occurrence

According to *Diagnosis and Treatment of Venous Thromboembolism during Pregnancy and Puerperium* [11], the occurrence of VTE in the study group was evaluated, namely, deep venous thrombosis and pulmonary embolism.

### 2.5. Observation Targets

(1) The platelet function-related indices of the study group and the control group were compared. (2) The patients in the study group were divided into a severe group, mild group, and nonbleeding group according to the severity of postpartum hemorrhage [9] to analyze the value of combination of platelet function-related indicators in evaluating the severity of postpartum hemorrhage in patients. (3) According to the occurrence of VTE, the patients in the study group were divided into a VTE group and non-VTE group to analyze the value of combination of platelet function-related indicators in predicting the occurrence of VTE in patients.

### 2.6. Statistical Process

SPSS22 software was used to process the data. The counting data were expressed as % and compared by the *χ*^2^ test between groups. The measurement data were expressed by $\bar{x}\pm S$ after the normal test and compared by *t*-test between groups. The ROC curve was used to analyze the value of platelet function in evaluating the severity of postpartum hemorrhage. The Spearman test was used to analyze the correlation between platelet function and severity of postpartum hemorrhage. *P* < 0.05 indicated that the difference was statistically significant.

## 3. Results

### 3.1. Comparison of Platelet Function between the Study Group and Control Group

The PLT value of the study group was lower than that of the control group, while PDW and MPV values were higher than those of the control group (all *P* < 0.05, Figure 1).

### 3.2. Comparison of Platelet Function between the Severe Group, Mild Group, and Nonbleeding Group

The patients in the study group were divided into the severe group (*n* = 13), mild group (*n* = 28), and nonbleeding group (*n* = 52) according to the severity of postpartum hemorrhage. PLT increased with the aggravation of postpartum hemorrhage, while PDW and MPV decreased with the aggravation of postpartum hemorrhage (all *P* < 0.05, Figure 2).

### 3.3. Value of Platelet Function in Evaluating the Severity of Postpartum Hemorrhage

The AUC of PLT, PDW, and MPV combination to evaluate the severity of postpartum hemorrhage in patients with gestational hypertension combined with diabetes was greater than that of PLT and PDW alone (both *P* < 0.05, Table 2 and Figure 3).

### 3.4. Correlation Analysis of Platelet Function and Severity of Postpartum Hemorrhage

PLT values were negatively correlated with the severity of postpartum hemorrhage, while PDW and MPV values were positively correlated with the severity of postpartum hemorrhage (all *P* < 0.05, Figure 4).

### 3.5. Comparison of Platelet Function between the VTE group and non-VTE group

The PLT value in the VTE group was higher than that in the non-VTE group, while PDW and MPV values were lower than those in the non-VTE group (all *P* < 0.05, Figure 5).

### 3.6. Predictive Value of Platelet Function on VTE in Patients with Gestational Hypertension and Diabetes Mellitus

The AUC of PLT, PDW, and MPV combination to predict the occurrence of VTE in patients with gestational hypertension combined with diabetes was greater than that of each index alone (*P* < 0.05, Table 3 and Figure 6).

## 4. Discussion

Gestational hypertension, as a common complication of pregnancy, usually occurs in the 20th week of pregnancy and later and is one of the main causes of maternal and perinatal death. Clinically, it is believed that the small blood vessel spasm throughout the body in the patients with gestational hypertension aggravates vascular endothelial injury, resulting in increased vascular permeability and fluid exudation, which in turn induces activation of coagulation factors and a hypercoagulable state of the body. Relevant reports indicate that the blood of pregnant women with pregnancy complications is mostly in a hypercoagulable state [12, 13]. Blood pressure is closely related to blood glucose level. In T2DM patients with hyperglycemia, glycation products in the body will increase subcutaneous collagen crosslinking, aggravating vascular wall fibrosis and increasing vascular wall stiffness, ultimately leading to hypertension. GDM not only causes complications such as abnormal amniotic fluid volume, premature rupture of membranes, and premature delivery but also leads to pregnancy outcomes such as neonatal asphyxia and hypoglycemia, seriously threatening the life and health of newborns. The blood of healthy pregnant women is also in a high coagulation state, which can effectively promote rapid and effective hemostasis after delivery. Moreover, the coagulation and fibrinolytic system are in a dynamic balance, which is conducive to the removal of microthrombus in the blood vessels and the promotion of endometrial regeneration and repair. Impaired glucose metabolism in patients with GDM can lead to vascular endothelial injury, resulting in platelet activation, enhanced coagulation function, weakened fibrinolysis and anticoagulation function, and changes in hemorheology and blood lipid levels. It is easy to aggravate the prethrombotic state, increase the risk of vascular disease or thrombosis, and cause medium- and long-term complications. Some studies have found that the probability of pregnancy-induced hypertension in GDM patients is much higher than that in normal women [14], suggesting that there may be a connection between the occurrence of the two diseases. Some scholars have found that platelet activation significantly enhanced fibrinolytic activity in patients with GDM, indicating that patients are in a state of hypercoagulability [15]. Platelets are generated by bone marrow megakaryocytes and participate in the coagulation process of the body. PLT and MPV reflect the number and average volume of platelets, respectively, and PDW reflects the degree of platelet volume difference. Pregnant women are prone to thrombocytopenia, and the probability of thrombocytopenia is about 11.6%. This study found that the PLT value of the study group was lower than that of the control group, while the PDW and MPV values were higher than those of the control group, indicating that abnormal platelet function existed in patients with gestational hypertension complicated with diabetes. This was mainly because vasospasm in patients caused vascular endothelial injury, peripheral blood platelet aggregation, and destruction, leading to thrombocytopenia, which stimulated the hematopoietic function of bone marrow and promoted the thrombopoiesis, thus resulting in the emergence of a large number of new large platelets in peripheral blood, which increased PDW and MPV values. Moreover, long-term hyperglycemia in GDM patients with hypertension damages vascular endothelial cells and the anticoagulant system, activates the coagulation system, and increases blood coagulation. In addition, abnormal glucose and lipid metabolism in patients can lead to changes in platelet membrane dynamics, thereby exposing membrane surface receptors, enhancing platelet adhesion and aggregation, and affecting platelet function in the body. The level of PLT decreased gradually in the hypertensive group, mild preeclampsia group, and severe preeclampsia group [16, 17].

Postpartum hemorrhage is the main cause of maternal death in China, and weakness of uterine contraction is the common cause. Most patients showed postpartum vaginal bleeding, hypotension, and other symptoms. Postpartum hemorrhage has great risk, so its prevention and early diagnosis are of great significance. Postpartum hemorrhage is a manifestation of coagulation dysfunction caused by the consumption of a large number of clotting substances and activation of the fibrinolytic system [18]. For now, relevant reports indicate that postpartum hemorrhage is closely associated with abnormal coagulation function [19, 20]. Platelet function is an important factor affecting the coagulation function of the body. It can realize hemostasis by releasing vasoconstrictor and clumping of platelets, which blocks damaged blood vessels and promotes coagulation. Related studies have found that thrombocytopenia is a risk factor for postpartum hemorrhage [21]. We conducted a retrospective study. The results of this study showed that PLT value was negatively correlated with the severity of postpartum hemorrhage, while PDW and MPV values were positively correlated with the severity of postpartum hemorrhage, indicating that the severity of postpartum hemorrhage was correlated with platelet dysfunction, further confirming the above view. Further study found that the AUC of the combination of platelet function-related indicators in evaluating the severity of postpartum hemorrhage in patients with gestational hypertension combined with diabetes was greater than 0.8, suggesting that the combination of platelet function-related indicators had a certain value in assessing the severity of postpartum hemorrhage. Therefore, the risk of severe postpartum hemorrhage can be predicted by detecting platelet function-related indicators. It is helpful for early clinical intervention and may reduce the incidence of severe postpartum bleeding.

VTE refers to abnormal coagulation of blood through deep veins, resulting in vascular blockage and blocked blood flow, which will not only affect patients' limb activities but also cause pulmonary embolism once the thrombus falls off, endangering patients' lives [22–24]. During pregnancy and puerperium, due to the factor such as activity reduction, postpartum physical recovery, and anesthesia, the blood flow rate of the body is easy to slow down, which can induce VTE. VTE can lead to spasm of small blood vessels throughout the body, resulting in reduced blood perfusion in all organs including the placenta as well as placental dysfunction, while the fetus is in a long-term ischemia and hypoxia environment, resulting in adverse pregnancy outcomes [25, 26]. Complications during pregnancy can aggravate the body's blood hypercoagulation and reduce the blood volume of effective circulation in the maternal body, leading insufficiency of blood perfusion in tissues and organs and damage of blood vessel cells, thus increasing the risk of VTE [27]. Currently, it is believed that the occurrence of VTE is closely related to the abnormal coagulation function of the body, suggesting that VTE patients may be accompanied by abnormal platelet function [28–30]. The above results of the present study showed that PDW and MPV values were significantly increased in patients with GDM combined with hypertension, indicating increased platelet activation and enhanced coagulation activity in vivo, showing increased possibility of thrombosis in patients. It was found in this study that the PLT value of the VTE group was higher than that of the non-VTE group, while the PDW and MPV values were lower than those of the non-VTE group, indicating that there was abnormal platelet function in VTE patients, mainly because of the fact that abnormal platelet function could lead to significant changes in the coagulation function and anticoagulant function of patients. This study also found that the combination of PLT, PDW, and MPV had predictive value on VTE occurrence in patients with both gestational hypertension and diabetes mellitus. This is mainly because the platelet abnormalities could increase the body high coagulation state and lead to vascular injury and the circulation of the blood stasis, which were direct risk factors for VTE occurrence. Patients with platelet dysfunction will have greatly increased risk of VTE. At present, many studies focus on platelet function in pregnant patients. However, few scholars have studied the relationship between platelet function and gestational hypertension combined with diabetes, which is also the innovation of this study.

In conclusion, abnormal platelet function existed in patients with gestational hypertension combined with diabetes, and platelet function was related to postpartum hemorrhage and the occurrence of VTE. In this study, abnormal platelet function was found in patients with gestational hypertension complicated with diabetes, and platelet function was related to postpartum hemorrhage and the occurrence of VTE. This suggests that patients with gestational hypertension and diabetes should pay more attention to abnormal platelet function. If abnormal platelet function occurs, postpartum hemorrhage and the risk of VTE should be anticipated. Deficiency still existed in this study. Only 93 patients were included for analysis. Too small sample size may lead to bias in the study results, so larger sample size is needed for further analysis in the later stage to ensure the accuracy of the study results.

## Figures and Tables

**Figure 1:** Comparison of platelet function between the study group and control group. Note: comparison of PLT, PDW, and MPV values between the two groups (^∗^*P* < 0.05).

**Figure 2:** Comparison of platelet function between the severe group, mild group, and nonbleeding group. Comparison of PLT, PDW, and MPV among the three groups (*P* < 0.05).

**Figure 3:** Value of platelet function in evaluating the severity of postpartum hemorrhage.

**Figure 4:** Correlation analysis of platelet function and severity of postpartum hemorrhage.

**Figure 5:** Comparison of platelet function between the VTE group and non-VTE group. Note: comparison of PLT, PDW, and MPV values between the two groups (^∗^*P* < 0.05).

**Figure 6:** ROC curve analysis of platelet function in predicting VTE in gestational hypertension with diabetes mellitus.

**Table 1:** Comparison of general data between the study group and control group.

Classification	Study group (*n* = 93)	Control group (*n* = 56)	*t* value	*P* value
Age (years)	27.68 ± 4.20	28.73 ± 4.08	1.494	0.137
Body mass index (kg/m^2^)	25.11 ± 1.66	25.44 ± 1.47	1.226	0.222
Pregnancy times (times)	1.69 ± 0.47	1.61 ± 0.49	0.990	0.324
Production times (times)	0.85 ± 0.36	0.88 ± 0.33	0.508	0.612
Gestational week (weeks)	35.22 ± 3.15	35.43 ± 2.21	0.438	0.662
Fasting blood glucose (mmol/L)	7.40 ± 1.01	4.32 ± 1.25	16.508	<0.001
Postprandial blood sugar (mmol/L)	12.12 ± 2.08	8.86 ± 1.98	8.539	<0.001
Glycosylated hemoglobin (%)	7.68 ± 0.93	5.97 ± 0.82	11.373	<0.001
Diastolic blood pressure (mmHg)	93.72 ± 5.11	84.00 ± 5.45	10.991	<0.001
Systolic blood pressure (mmHg)	149.54 ± 8.85	125.95 ± 11.16	14.300	<0.001

**Table 2:** Value of platelet function in evaluating the severity of postpartum hemorrhage.

Group	Cutoff value	AUC	SE	95% CI
PLT	183.87∗10^9^/L	0.706^∗^	0.105	0.500~0.912
PDW	18.04%	0.749^∗^	0.108	0.537~0.960
MPV	12.79 fl	0.816	0.080	0.659~0.973
Combination		0.852	0.078	0.700~1.000

Note: compared with combination (^∗^*P* < 0.05).

**Table 3:** Predictive value of platelet function on VTE in patients with gestational hypertension and diabetes mellitus.

Group	Cutoff value	AUC	SE	95% CI
PLT	207.14∗10^9^/L	0.718^∗^	0.070	0.581~0.854
PDW	15.95%	0.676^∗^	0.110	0.460~0.892
MPV	9.79 fl	0.787^∗^	0.059	0.672~0.901
Combination		0.890	0.037	0.817~0.963

Note: compared with combination (^∗^*P* < 0.05).

## Data Availability

The labeled dataset used to support the findings of this study are available from the corresponding author upon request.
